This article has been retracted.

# Protein Arginine Methyltransferase 5 Promotes the Migration of AML Cells by Regulating the Expression of Leukocyte Immunoglobulin-Like Receptor B4

**DOI:** 10.1155/2021/7329072

**Published:** 2021-10-19

**Authors:** Lu Zhao, Bingqing Cheng, Jie Xiong, Dan Ma, Xin Liu, Li Wang, Xi Zhang, Jishi Wang

**Affiliations:** ^1^School of Clinical Medicine, Guizhou Medical University, Guiyang 550004, China; ^2^Medical Center of Hematology, Xinqiao Hospital, State Key Laboratory of Trauma, Burn and Combined Injury, Army Medical University, Chongqing 400037, China; ^3^Department of Hematology, Affiliated Hospital of Guizhou Medical University, Guiyang 550004, China; ^4^Key Laboratory of Hematological Disease Diagnostic and Treat Centre of Guizhou Province, Guiyang 550004, China

## Abstract

Acute myeloid leukemia (AML) is the most common type of acute leukemia in adults with poor prognosis. Especially for AML-M5 type, due to the strong cell migration ability, the possibility of extramedullary invasion is large and widespread, which leads to poor therapeutic effect. Previous studies have found that protein arginine methyltransferase 5 (PRMT5) could promote the proliferation and differentiation of leukemic cells in AML, but its regulation on the invasive ability of AML cells remains unclear. This study was designed to explore the role of PRMT5 in regulating the invasion of AML cells and to investigate the mechanisms. Patient samples were collected for detection of PRMT5 expression level. AML cells were used for exploring the function of PRMT5. The results of clinical samples showed that the expression of PRMT5 was significantly increased in newly diagnosed and recurrent AML patients, and the expression of leukocyte immunoglobulin-like receptor B4 (LILRB4) was positively correlated with the level of PRMT5. In the cell experiment in vitro, we found that when PRMT5 was knocked down, the invasion, migration, and adhesion capacities of MV-4-11 cells and THP-1 cells were decreased, and the mRNA and protein levels of LILRB4 were also decreased. Moreover, we screened related signaling pathways and found that PRMT5 affected the expression of downstream LILRB4 by activating mTOR pathway, which in turn enhanced the invasive ability of AML cells. Taken together, PRMT5 plays an important role in the invasion of AML, which acts via regulating the expression of LILRB4. PRMT5 could act as a potential therapeutic candidate for AML.

## 1. Background

Acute myeloid leukemia (AML) is the most common type of acute leukemia in adults. Despite the various therapeutic discoveries on AML with the deepening research [1–4], the “anthracycline-cytarabine” regimen remains the commonly used chemotherapeutic regimen. AML is still definitely a catastrophic disease [1, 5–7]. In recent years, it has been proven that acute leukemia is often accompanied by extramedullary infiltration (EMI). The incidence of EMI in AML is approximately 20%-40%, mostly in M5 (acute monocytic leukemia) and M4 (acute myelomonocytic leukemia) types according to French-American-British (FAB) classification system. For the majority of these patients, the remission rate after induction chemotherapy is low, with poor prognosis [1, 8]. Therefore, it is of great significance to study the EMI mechanism of AML and to explore the therapeutic targets for AML.

Protein arginine methyltransferases (PRMTs) are a type of enzymes that transfer methyl from cofactor S-Adenosylmethionine (SAM) to substrate protein arginine omega-nitrogen. According to its specificity, PRMTs can be divided into three subgroups: I, II, and III, which are asymmetric dicarboxylic esters, symmetric dicarboxylic esters, and monomethylated substrates, respectively [9]. Protein arginine methyltransferase 5 (PRMT5), a kind of type II PRMT, catalyzes the symmetrical dimethylation of protein arginine residues, which is involved in diverse cellular processes, including transcription, DNA damage response, splicing, translation, and cellular signal transduction [10, 11]. Some studies have shown that PRMT5 is not only involved in the development of normal human immune system, but also participates in the regulation of tumor invasion, migration, and T cell-mediated immune response as well as pathological process of AML [12–15]. The overexpression of PRMT5 is detected in various types of AML cell lines [10, 16, 17]. Functionally, PRMT5 can inactivate p53 by methylation, affect mixed lineage leukemia rearrangement, or promote the growth of leukemia through microRNA (miR)/protein network, thereby promoting cell differentiation and proliferation [17–20]. In addition, PRMT5 can alter the transcriptional process of multiple essential genes through the methylation of splice regulators, which is necessary to maintain the survival of leukemic cells [16, 17, 21, 22]. Therefore, suppressing PRMT5 represents an exciting anticancer strategy. At present, three types of PRMT5 inhibitors are available to treat solid cancers and blood malignancies. However, the role of PRMT5 in AML has not been completely clarified, and the role and mechanism of PRMT5 in tumor invasion and migration also remain unclear.

Leukocyte Ig-like receptor subfamily B (LILRB) is a group of type I transmembrane glycoproteins with ligand-bound extracellular Ig-like domain and intracellular immune receptor tyrosine inhibitory motif (ITIMs) and can recruit tyrosine phosphatase SHP-1, SHP-2, or inositol phosphatase SHIP, with immunosuppressive function [23–26]. Thus, leukocyte immunoglobulin-like receptor B4 (LILRB4) is considered as an immune checkpoint protein [27, 28]. Moreover, LILRB4 could act as a tumor maintenance factor, but it may not affect normal development, which is an attractive target for cancer treatment [26, 28, 29]. Monocyte AML is a subtype of AML. Extramedullary diseases, including gingival infiltration and involvement of skin and cerebrospinal fluid, are common in monocyte AML [28]. The latest findings show the low expression of LILRB4 in normal monocytes [24, 25] and high expression of LILRB4 in monocytes of acute monocytic leukemia, which is a marker of monocyte AML [30]. It can inhibit immune activation, promote tumor infiltration and invasion, and affect the invasive ability in AML [28, 29, 31]. Some studies have suggested that PRMT5 plays important roles in the regulation of immune response, migration, and invasion in tumorigenesis [12–15, 20]. In addition, PRMT5 can regulate the downstream factors of LILRB4 [31–33].

In this study, we investigated the changes of PRMT5 expression in AML-M5 patients, MV-4-11, and THP-1 and further explored the effects of PRMT5 on the invasion and migration in AML. Moreover, we also examined the correlation between PRMT5 and LILRB4 in relation with AML infiltration and additionally assessed the pathway underlying the effects of PRMT5 methylation on the expression of LILRB4, aiming to provide experimental evidence for the treatment of AML.

## 2. Methods and Materials

### 2.1. Patient Samples

Bone marrow samples were collected from 30 (AML-M5 or AML-M4) patients from the Affiliated Hospital of Guiyang Medical University (Guiyang City, Guizhou Province) from May 2018 to April 2020 (Table 1). All AML samples were collected from bone marrow of untreated patients. In addition, 20 hematopoietic stem cell transplantation donors were collected from Guizhou hematopoietic stem cell laboratory as the normal control. All patients were diagnosed by FAB and confirmed by clinical laboratory examination, blood routine examination, and bone marrow examination. These AML samples were from bone marrow of untreated patients. And in all patient samples, the number of bone marrow blasts is ≥80%. We collected individual bone marrow nuclear cells from AML patients and the hematopoietic stem cell transplant donor by Ficoll gradient centrifugation. According to the Helsinki Declaration, AML patients who provided primary AML samples signed written informed consent. The study protocol was approved by the Medical Science Ethics Review Committee of the University Hospital of Guizhou Medical University (2019 Ethical Review No. 123).

### 2.2. Cell Culture

Human THP-1 (AML-M5), kasumi-1 (AML-M2), HL-60 (human promyelocytic leukemia cell), and MV-4-11 (AML-M4) cells were cultured in RPMI1640 medium and IMDM medium containing 10% fetal bovine serum (FBS), respectively. The primordial cells of patients with AML were taken from the blood samples of patients from the Affiliated Hospital of Guizhou Medical University and stored in the leukemia cell bank of the Affiliated Hospital of Guizhou Medical University. All cells were incubated at 37°C and 5% CO_2_.

### 2.3. Reagents and Antibodies

EPZ015666 and mTOR inhibitor-3 were purchased from MCE (China). Antibody against PRMT5 (YN3030) was purchased from Immunoway (Suzhou, China). Anti-LILRB4 (K004989P), anti-PI3K (K106692P), anti-phosph-PI3K (K006379P), anti-AKT (K101311P), anti-phosph-AKT (K006214P), anti-NF-*κ*B (K002162P), anti-phosph-NF-*κ*B (K006209P), anti-mTOR (K003351P), and anti-phosph-mTOR (K006205P) antibodies were purchased from Solei Bao Technology (Beijing). Anti-ERK (4695T) and anti-phosph-ERK(4370T) were purchased from Cell Signaling Technology (Danvers, MA, USA).

### 2.4. Western Blot Analysis

After washing with saline twice, cells were lysed in RIPA buffer containing PMSF and proteasome inhibitor to extract the total protein (Solarbio Life Sciences Technology Co., Ltd., Beijing, China), followed by quantification of protein concentration by BCA protein concentration assay kit (Solei Bao Technology Co., Ltd., Beijing, China). The same amount of protein (20 *μ*g) was separated by 10% SDS-PAGE gel and transferred to the PVDF membrane (Millipore Company, Milford, Massachusetts, USA). Membranes were subsequently blocked with 5% skim milk diluted in TBST for 2 h and incubated with primary antibody (1 : 1000) overnight, followed by incubation with fluorescent coupled secondary antibody (1: 2000). *β*-Actin was used as the loading control and for normalization. The signal strength of the film was measured by Tanon (Shanghai, China).

### 2.5. RT-qPCR

Total RNA was extracted from MV-4-11, THP-1, and bone marrow blood samples of patients by the Trizol method. Afterwards, reverse transcription was performed with Single strand cDNA synthesis kit. qRT-PCR was performed using an SYBR Green PCR Master Mix (TianGen Biotech, Beijing, China) and a PRISM 7500 real-time PCR detection system (ABI, USA). The expression level of target gene was normalized to that of *β*-actin. The primer sequences for qRT-PCR were as follows: PRMT5F: 5′-GGGAAGAGGATGGGAAAC-3′ and PRMT5R: 5′-TGATTGACAACAACCGCTAT-3′; LILRB4F: 5′-TCAGTACCTCCCAGTGCC-3′ and LILRB4R: 5′-CCACAAGGTCCGTCTCAA-3′; and *β*-actinF: 5′-CTACCTCATGAAGATCCTCACCGA-3′ and *β*-actinR: 5′-TTCTCCTTAATGTCACGCACGATT-3′.

### 2.6. Small Interference with RNA-Transfected Cells

siRNA against PRMT5 (si-PRMT5) was used to suppress the expression of PRMT5 in cells. Sasastic siRNA (si-NC) was used as the negative control. The siRNA sequence was designed and synthesized by Quan yang Biotechnology Co., Ltd. (Shanghai, China).

The sequence is as follows: si-PRMT5: 5′-GGGACUGGAAUACGCUAAUTT—3′.

The final concentration per siRNA was 2.5 nmol. According to the commodity specification, Lipo8000TM transdye reagent and siRNA raw solution (250 *μ*l/hole) were mixed and further added to the ThP-1 and MV-4-11 cells, followed by incubation for 48 h. Western blot was used to detect the downregulation efficiency of siRNA.

### 2.7. Transwell Migration and Invasion Assay

siRNA was used to downregulate the expression of PRMT5 in MV-4-11 and THP-1 cells, followed by assessment of the migration and invasion ability of the corresponding cells. In brief, leukemia cells (5 × 10^4^ cells/ml) were added to the polycarbonate membrane (pore size 8 *μ*m, BD Biosciences) for migration assay and polycarbonate membrane with fibronectin coating (pore size 8 *μ*m, BD Biosciences) for invasion assay, respectively, and 600 *μ*l RPMI1640 medium was added to the lower chamber of Transwell. After incubation at 37°C for 24 h, cells were observed under microscope (100x) by randomly selecting nine views from each well, aiming to count the number of cells penetrating into the lower cavity and to observe cell morphology.

### 2.8. Cell Adhesion Assay

In order to study the effect of PRMT5 on the adhesion ability of leukemic cells, Beibo Cell Adhesion Test Kit (Bestbio, China) was purchased to detect the cell adhesion ability of THP-1 and MV-4-11 cells after downregulating PRMT5 and the corresponding control cells at the same time. Briefly, 100 *μ*l/well coating solution was added to the 96-well plate at 4°C overnight. After washing with PBS twice, 5 × 10^4^/ml cells per well were inoculated and incubated at 37°C for 1 h. Afterwards, 10 *μ*l staining solution of 37°C was added and incubated for additional 2-4 h, followed by detection of the absorbance of 450 nm by enzyme labeling instrument.

### 2.9. Statistical Analysis

All results were analyzed using the GraphPad Prism 7.0 software. Data were presented as mean ± SD and analyzed by either one-way ANOVA or Student's *t*-test. *P* < 0.05 was considered as statistically significant.

## 3. Results

### 3.1. The High Expression of PRMT5 in AML-M5 Patients

Blood samples from 30 patients with AML-M5 or AML-M4 and 20 normal controls were collected from the Hematopoietic Stem Cell Laboratory of the Affiliated Hospital of Guizhou Medical University from May 2018 to April 2020. The clinical characteristics of the patients are summarized in Table 1. RT-qPCR analysis revealed the expression of PRMT5 in AML patients. As a result, the mRNA expression of PRMT5 was the highest in the recurrent group, sequentially followed by the newly diagnosed group and normal control group (Figure 1(a)). Similarly, RT-qPCR was used to detect the expression of LILRB4 in AML patients, and the mRNA expression of LILRB4 was significantly higher in AML patients than that in normal subjects (Figure 1(b)). Patients were divided into primary diagnosis group and recurrence group. The mRNA expression of LILRB4 was significantly higher in recurrent patients than that in the primary diagnosis group (Figure 1(b)). In addition, the protein levels of PRMT5 and LILRB4 were detected by Western blot, which was consistent with those of RT-qPCR (Figure 1(c)). The protein levels of PRMT5 and LILRB4 were the highest in recurrent patients, followed by newly diagnosed patients and normal control (Figures 1(d) and 1(e)). These results indicated that the expressions of PRMT5 and LILRB4 were increased in AML patients, especially in recurrent patients.

In order to determine whether PRMT5 was closely correlated with LILRB4, we investigated the correlation coefficient. Log_10_^*X*^ was used to calculate the mRNA level of PRMT5 and LILRB4. According to the *R* value, there was a positive correlation between PRMT5 and LILRB4 (Figure 1(f)), suggesting the positive correlation between the expression of PRMT5 and LILRB4 in AML patients.

### 3.2. The Changes in Migration, Invasion, and Adhesion of AML Cells after Downregulating PRMT5

We detected the expression of PRMT5 in AML cell lines (THP-1, MV-4-11, kasumi-1, and HL-60) and normal human samples by Western blot. As a result, the expression of PRMT5 in cell lines was higher than in normal human samples (Figure 2(a)). Moreover, the expression of PRMT5 in THP-1 and MV-4-11 cell lines was higher than that in other cell lines. Grayscale analysis of all Western blot bands showed the significantly high expression of PRMT5 in THP-1, MV-4-11, and kasumi-1 than normal human samples. And PRMT5 expression was the highest in THP-1 and MV-4-11 (Figure 2(b)). Therefore, THP-1 and MV-4-11 were selected for subsequent experiments.

Although the increased expression of PRMT5 has been confirmed to be associated with the pathogenesis and prognosis of AML and to affect the proliferation and differentiation of AML cells, however, the effects of PRMT5 on the invasion and migration of AML cells were not well-studied. To confirm the roles of PRMT5 expression in the adhesion, invasion, and migration of AML cells, we assessed the adhesion, invasion, and migration abilities of MV-4-11 (Figure 2) and THP-1 (Figure 3) cells after downregulation of PRMT5 expression. siRNA was used to downregulate the expression of PRMT5 in AML cells, followed by assessment of the suppressed expression of PRMT5 by Western blot and RT-qPCR (Figures 2(c) and 3(b)). Afterwards, we examined the effects of PRMT5 expression on cell adhesion and found that the adhesion ability of cells was significantly decreased in the si-PRMT5 group (Figures 2(d) and 3(b)). Observation of cell morphology revealed that the morphological integrity of cells in the si-PRMT5 group was worse than that in the CON group, and the number of malformed cells in the si-PRMT5 group was significantly more than that in the CON group (Figures 2(e) and 3(c)). Transwell assay was used to detect the migration ability of the treated cells, indicating that the migration ability of the two AML cell lines in the si-PRMT5 group was significantly lower than that in the CON group (Figures 2(f) and 3(d)). We further evaluated the changes of cell invasion that were consistent with the migration assay. The number of cells infiltrating from the upper chamber to the lower chamber in the si-PRMT5 group was significantly less than that in the CON one (Figures 2(g) and 2(h) and 3(e) and 3(f)).

To further validate the results, PRMT5 inhibitors (EPZ015666) were purchased to inhibit PRMT5 expression in MV-4-11 and THP-1 cells. And Western blot was used to detect PRMT5 expression in MV-4-11 and THP-1 cells, showing that the expression of PRMT5 in the EP015666 group was significantly decreased (Figures 4(e) and 4(i)). We further examined the migration, invasion, and adhesion abilities and morphology of THP-1 and MV-4-11 cell lines after the treatment of PRMT5 inhibitors. Based on the experimental results of MV-4-11 cells, we observed that the morphology of the cells penetrating the membrane pore after PRMT5 inhibition was worse than that of the CON group, and the cell fragments increased (Figure 4(a)). The number of cell migration in the PRMT5 inhibitor group was significantly decreased compared with that in the CON group (Figure 4(b)). Consistent with migration analysis, invasion assay revealed the similar results. (Figures 4(c) and 4(d)). Moreover, after the administration of PRMT5 in MV-4-11, the adhesion ability of AML cells was also inhibited (Figure 4(f)), which was consistent with the results after PRMT5 downregulation in MV-4-11. Similar observations were also detectable from THP-1 cells (Figures 4(g)–4(l)). Taken together, these results revealed that the expression of PRMT5 affected cell adhesion, migration, and invasion of AML cells.

### 3.3. PRMT5 Downregulation Decreases the Expression of LILRB4

In order to verify whether PRMT5 affected the invasiveness of AML cells by downregulating the expression of LILRB4, protein samples were extracted from AML cells after downregulating PRMT5. As a result, the expression of LILRB4 was significantly lower in the si-PRMT5 group than in the CON group of MV-4-11 cells (Figure 5(a)), and the grayscale analysis showed that the downward adjustment was statistically significant on both (Figures 5(b) and 5(c)). Similar findings were also detected on THP-1 cells (Figures 5(d)–5(f)). Thus, the expression of LILRB4 was decreased following downregulation of PRMT5 in AML cells.

### 3.4. PRMT5 Knockdown Affects AKT, ERK, and mTOR Pathways in AML Cells

Previous studies have shown that PRMT5 is involved in the regulation of AKT, ERK, NF-*κ*B, and mTOR pathways [34]. Silencing of PRMT5 can lead to the inhibition of AKT and ERK pathways, which in turn inhibit mTOR pathway [35], thus affecting the apoptosis and migration of lung cancer [19]. To determine whether PRMT5 affected the expression of LILRB4 and the invasiveness of AML cells through relevant pathways, MV-4-11 cells with downregulation of PRMT5 were extracted and subjected to Western blot. Compared with the CON group and si-CN one, the phosphorylation of AKT, mTOR, and ERK pathways was inhibited in si-PRMT5 groups of both MV-4-11 (Figure 6(a)) and THP-1 cells (Figure 6(c)), while the phosphorylation of NF-*κ*B pathway was only affected in THP-1 (Figure 6(d)) but not MV-4-11 (Figure 6(b)) cells. Thus, PRMT5 knockdown by siRNA significantly decreased the phosphorylation of AKT, mTOR, and ERK pathways in AML cell lines of both MV-4-11 and THP-1 cells.

### 3.5. Blocking mTOR Pathway Affects the Expression of LILRB4 and Invasion, Migration, and Adhesion of AML Cells

Since AKT/mTOR and ERK/mTOR pathways were significantly affected after the downregulation of PRMT5 in AML cell lines, we speculated that PRMT5 might affect the expression of LILRB4 and the invasive capability of AML cells through AKT/mTOR and ERK/mTOR axes. Thus, we applied an inhibitor of mTOR pathway, mTOR inhibitor-3, on both MV-4-11 and THP-1 cell lines, followed by examination of both morphology and migration, invasiveness, and adhesion. As the results yielded from the experiments of MV-4-11 cells, we observed that not only the morphology (Figure 7(a)) of the cells infiltrating through the membrane barrier after inhibition of mTOR was worse than that of the CON group, with increased cell fragments, but also the migration (Figure 7(b)) of cells treated by mTOR inhibitor was significantly less. Consistent with migration assay, the invasion assay yielded similar results (Figures 7(c) and 7(d)). Additionally, the inhibition of the mTOR pathway also led to the suppressed adhesion ability of AML cells (Figure 7(e)), which was consistent with outcomes after the downregulation of PRMT5. Similar observations were also obtained from THP-1 cells (Figure 7(f)–7(j)).

To further validate the results, we used PRMT5 inhibitors (EPZ015666) to inhibit PRMT5 expression in both MV-4-11 and THP-1 cells. Western blot was used to detect the changes of mTOR pathway and LILRB4 at protein level in MV-4-11 (Figure 8(a)), which revealed that the phosphorylation of mTOR pathway was inhibited (Figure 8(d), *P* < 0.05) and the expression of LILRB4 was inhibited (Figure 8(e), *P* < 0.05). Meanwhile, we observed the same changes in THP-1 cell lines (Figures 8(b)–8(h)).

In order to explore the relationship between the above changes and LILRB4, we detected the proteins of PRMT5 and LILRB4 in AML cells after blocking mTOR pathway. Therefore, after blocking mTOR pathway, the protein abundance of LILRB4 in the mTOR inhibitor-3 group was significantly lower than that in the CON group of both MV-4-11 (Figure 9(a)) and THP-1 (Figure 9(b)) cells, which were statistically significant indicated by image gray analysis (Figures 9(c) and 9(d)). These results suggested that the expression of LILRB4 was regulated by the mTOR pathway.

## 4. Discussion

Some studies have shown that PRMT5 is necessary for the survival of AML cells and is highly expressed in many types of leukemia, especially in M5 leukemia [20, 37]. However, the pathogenesis of AML is complex, and little is known about the specific role of PRMT5 in AML. Inhibition of PRMT5 expression has been reported to functionally exert antitumor effects and can be used as a promising therapeutic target. It can induce alternative splicing changes of a variety of essential genes through the mysterious splicing regulatory factor SRSF1 [18, 21, 38].

PRMT5 exists in the nucleus and cytoplasm. A great deal of evidence shows that PRMT5 activates or suppresses the transcription via the methylation of arginine on histone and promotes cancer by inhibiting the expression of tumor suppressor gene [1, 9, 16, 17, 20]. PRMT5 is highly expressed in malignant hematological diseases such as leukemia and lymphoma and participates in the expression and regulation of many genes [17]. It is an important regulator of cell proliferation and differentiation, which has been attracting more and more attention. It is also involved in the regulation of proliferation and survival pathway, epigenetic regulation of anticancer target genes, and organelle biogenesis [20, 35–37]. Previous studies have shown that PRMT5 is overexpressed in many malignant tumors such as acute lymphoblastic leukemia and is closely related to tumor growth [16, 17]. Several studies have shown whether PRMT5 is essential for the survival of AML cells and its expression pattern in many types of leukemia, especially in M5 leukemia [20, 37]. In this study, the effects of PRMT5 on the invasion and migration in AML cells were investigated. Firstly, the clinical samples from 30 AML-M5 patients were examined, showing that the expression of PRMT5 was high in AML-M5 patients, and the expression of PRMT was significantly higher in recurrent patients than that in other patients, indicating that the overexpression of PRMT5 was associated with the recurrence of AML (Figure 1). AML-M5 is more prone to present EMI and recurrence than other types of leukemia. According to this phenomenon, PRMT5 expression is associated with specific types of leukemia and is correlated with the invasive ability of tumor. Moreover, we found that PRMT5 was highly expressed in AML cell lines, and the expression of PRMT5 in MV-4-11 and THP-1 was higher than kasumi-1 and HL-60 (Figures 2(a) and 2(b)). The effects of PRMT5 on the invasion and migration of AML were investigated in MV-4-11 and THP-1. siRNA and EPZ015666 inhibitor were used to inhibit PRMT5 expression. The capability of migration, invasion, and adhesion of THP-1 and MV-4-11 was significantly decreased (Figures 2–4). These results have shown that PRMT5 plays important roles in invasion and migration in AML-M5.

Recent studies have shown that LILRB4 is vitally involved in the pathogenesis and development of AML, and the overexpression of LILRB4 in AML-M5 is closely associated with the invasive ability of AML-M5 [26]. We further examined the expression of LILRB4 in 30 patients and found that the expression of LILRB4 in patients was higher than that in normal subjects. The expression of LILRB4 was the highest in recurrent patients (Figure 1(b)) and positively correlated with PRMT5 (Figure 1(f)), suggesting that LILRB4 may be involved in the pathogenesis of AML. There may be a certain relationship between PRMT5 and LILRB4 in regulating the invasion and migration of AML. This result is consistent with the characteristics of AML in previous studies [29], and our results further confirm that the overexpression of PRMT5 is closely associated with the expression of LILRB4 in highly invasive AML. In addition, our results provide evidence that the expression of LILRB4 is significantly decreased after downregulation of PRMT5. Meanwhile, the capability of invasion, migration, and adhesion in AML cells is also significantly decreased, similar to that following downregulation of LILRB4 expression [29]. Thus, PRMT5 may affect the invasion and migration of AML by regulating the expression of LILRB4.

In addition, the mechanism underlying the effects of PRMT5 on downstream gene expression and phenomena was also discussed. To be specific, in lung cancer, inhibition of PRMT5 expression can alleviate the trigger of enolase-1, thus reducing the invasion of lung adenocarcinoma [38]. Previous studies have also shown that PRMT5 can regulate PI3K, AKT, ERK, mTOR, and NF-*κ*B signaling pathway [16, 17, 20, 34]. PRMT5 affects the expression of multiple essential genes by regulating splicing [21]. In this study, we selected several approaches and found that the change of mTOR pathway was the most significant. Strobl et al. have found that the inhibition of PRMT5 is consistent with the induction of p53 expression and the decrease of AKT/mTOR signal transduction in lung cancer [19]. Wei et al. have found that PRMT5 affects the apoptosis and invasion of lung cancer cells by regulating the expression of AKT/mTOR or ERK/mTOR [34]. These results suggest that PRMT5 plays a biological role in AML through the mTOR pathway. In this study, downregulation of PRMT5 was used to inhibit the expression of LILRB4, which further decreased the invasive ability of THP-1 and MV-4-11 cells. We speculated that PRMT5 might affect the expression of LILRB4 by activating AKT/mTOR and ERK/mTOR axes. Therefore, mTOR inhibitors were used to suppress the phosphorylated expression of mTOR pathway, followed by detection of downstream phenomena and LILRB4 expression. These results showed that the expression of LILRB4 was significantly decreased, and the migration, invasion, and adhesion abilities of THP-1 and MV-4-11 were significantly decreased. The above findings indicate that the expression of LILRB4 is inhibited under suppressed mTOR phosphorylation. PRMT5 is the upstream gene of LILRB4 and regulates the expression of LILRB4 through mTOR pathway, thus affecting the invasive ability of AML.

## 5. Conclusions

PRMT5 is highly expressed in AML, which is a marker of poor prognosis for AML. PRMT5 plays an important role in the invasive capability of AML cells. Inhibition of PRMT5 can alleviate the invasion and migration of AML cells and improve the prognosis of AML, which is associated with the change of LILRB4 induced by PRMT5. The effects of PRMT5 on LILRB4 may be associated with its regulation on mTOR. The overexpression of PRMT5 is critically involved in the invasion and migration of AML, which could act as a new therapeutic target for AML.

## Figures and Tables

**Figure 1:** Real-time qPCR and Western blot analyses of the levels of PRMT5 and LILRB4 in 30 patients with AML-M5. The mRNA levels of (a) PRMT5 and (b) LILRB4 were detected by real-time qPCR in normal subjects, newly diagnosed patients, and recurrent ones. (c) Western blot analysis was performed to detect the protein abundances of PRMT5 and LILRB4 (normal persons, *n* = 2; newly diagnosed cases, *n* = 2; and recurrent cases, *n* = 2). *β*-Actin was used as the internal control. Western blot and subsequent grayscale analysis revealed that the expression of (d) PRMT5 and (e) LILRB4 was higher in the relapse group than that in the newly diagnosed group. (f) The analysis of correlation coefficient indicated that the expression of PRMT5 was positively correlated with that of LILRB4 (*r* = 0.8215, *P* ≤ 0.0001). Each value was presented as log_10_^*X*^. All the experiments were repeated in triplicates. The data are expressed by mean ± standard deviation (^∗^*P* ≤ 0.05; ^∗∗^*P* ≤ 0.01). The 2-*Δ* CT method was used for quantitative presentation of relative mRNA levels. The error bar represents ±SD (^∗^*P* ≤ 0.05; ^∗∗^*P* ≤ 0.01; ^∗∗∗^*P* ≤ 0.001; ^∗∗∗∗^*P* ≤ 0.0001).

**Figure 2:** Detection of expression in human samples and AML cell lines. (a) Western blot was used to detect the protein level expression in PRMT5 (normal, THP-1, MV-4-11, kasum-1, and HL-60), respectively. *β*- Actin was used as the internal control. (b) Western blot and subsequent grayscale analysis revealed the expression of PRMT5. Downregulation of PRMT5 gene by siRNA could inhibit the migration, invasion, and adhesion of MV-4-11. (c) PRMT5 silencing by siRNA on AML. After treatment with si-PRMT5 or NC siRNA for 48 h, the expression of PRMT5 in protein (upper) and mRNA (lower) level was significantly decreased in MV-4-11 cells. (d) Adhesion assay exhibited that the adhesion capability of MV-4-11 cells in the si-PRMT5 group was significantly lower than that in the wild type group and si-CN group. (e) Transwell assay was performed to detect the migration of MV-4-11 cells in the wild type group, si-CN group, and si-PRMT5 group. (f) Quantitative analysis of the number of migrating cells in each group after 24 h indicated that the number of migrating cells in the si-PRMT5 group was significantly decreased. (g) After downregulation of PRMT5 by siRNA, the invasion of MV-4-11 cells in each group was observed. (h) Quantitative analysis revealed that the number of invasion in MV-4-11 cells was significantly decreased. Data are expressed by mean ± standard deviation (^∗^*P* ≤ 0.05; ^∗∗^*P* ≤ 0.01; ^∗∗∗^*P* ≤ 0.001). The 2-*Δ* CT method was used for quantitative presentation of relative mRNA levels. The error bar represents ±SD. (^∗^*P* ≤ 0.05). The images of (c, e) are under 100x magnification.

**Figure 3:** Downregulation of PRMT5 gene by siRNA can inhibit the migration, invasion, and adhesion of THP-1. (a) After treatment with si-PRMT5 or NC siRNA for 48 h, the expression of PRMT5 in protein (upper) and mRNA (lower) level was significantly decreased in THP-1 cells. (b) Adhesion assay revealed that the adhesion capability of THP-1 cells in the si-PRMT5 group was significantly decreased than that in the wild type group and si-CN group. (c) Transwell assay was used to detect the migration of THP-1 cells in the CON group, si-CN group, and si-PRMT5 group. (d) Quantitative analysis of the number of migrating cells in each group after 24 h indicated that the number of migrating cells in the si-PRMT5 group was significantly decreased. (e) Invasion assay was performed to detect the migration of THP-1 cells in the CON group, si-CN group, and si-PRMT5 group. (f) Quantitative analysis of the number of invasion cells in each group after 24 h indicated that the number of invasion cells in the si-PRMT5 group was significantly decreased. All the experiments were performed in triplicate. Data are expressed by mean ± standard deviation (^∗^*P* ≤ 0.05; ^∗∗^*P* ≤ 0.01). 2-*Δ* CT was used for quantitative presentation of relative mRNA levels. The error bar represents ±SD (^∗∗^*P* ≤ 0.01). The images of (c, e) are under 100x magnification.

**Figure 4:** PRMT5 inhibitor (EPZ015666) attenuates the migration, invasion, and adhesion of AML cells. (a) After EPZ015666 treatment in MV-4-11 cells for 24 h, the numbers of cell migration in the CON group and EPZ015666 group were detected by Transwell migration study. (b) Quantification analysis of (a) indicated that the number of cells in the inhibitor group was significantly less than that in the CON group. (c) After EPZ015666 treatment in MV-4-11 cells for 24 h, the number of cell invasion in the CON group and inhibitor group was detected by Transwell invasion assay. (d) Quantification analysis of (c) indicated that the number of invasion cells in the inhibitor group was significantly less than that in the CON group. (e) After EPZ015666 treatment in MV-4-11 cells for 24 h, the protein expression of PRMT5 was changed. (f) After EPZ015666 treatment in MV-4-11 cells for 24 h, cell adhesion was detected, and the number of adherent cells in the inhibitor group was found to be significantly less than that in the CON group. After EPZ015666 treatment in THP-1 cells for 24 h, the (g, h) migration, (j, k) invasion, and (l) adhesion of THP-1 cells were detected. The above indexes in the inhibitor group were significantly lower than those in the CON group. (i) After EPZ015666 treatment in THP-1 cells for 24 h, the protein level of PRMT5 was changed. All the experiments were performed in triplicate. Data are expressed by mean ± standard deviation (^∗^*P* ≤ 0.05; ^∗∗^*P* ≤ 0.01). The representative images are under 100x magnification.

**Figure 5:** The effect of PRMT5 knockdown by siRNA on the protein abundance of LILRB4. (a) Western blot analysis of PRMT5 and LILRB4 protein in MV-4-11 cells of the CON group, si-CN group, and si-PRMT5 group after corresponding treatment for 48 h. *β*-Actin was used as the internal control. Subsequent grayscale analysis revealed the expression levels of (b) PRMT5 protein and (b) LILRB4 protein in MV-4-11 cells of the si-PRMT5 group were lower than those of other two groups. (d) Western blot analysis of PRMT5 and LILRB4 proteins in THP-1 cells of the CON group, si-CN group, and si-PRMT5 group after corresponding treatment for 48 h. *β*-Actin was used as the internal control. Subsequent grayscale analysis revealed that the expression levels of (e) PRMT5 protein and (f) LILRB4 protein in THP-1 cells of the si-PRMT5 group were lower than those of other two groups. All the experiments were repeated for three times. Data are expressed by mean ± standard deviation (^∗^*P* ≤ 0.05; ^∗∗^*P* ≤ 0.01).

**Figure 6:** The effect of PRMT5 knockdown by siRNA on several signaling pathways in AML cells. (a) Western blot was used to detect the changes of p/T-AKT, p/T-ERK, p/T-mTOR, p/T-NF-*κ*B, and p/T-PI3K in MV-4-11 cells after siRNA knockdown of PRMT5 gene. (*top*) Western blot images (*β*-actin as loading control); (*bottom*) image grayscale analysis of the corresponding Western blot images in triplicates. The results indicated that the expression levels of p-ERK, p-AKT, and p-mTOR were decreased in the si-PRMT5 group. (b) Western blot was used to determine the changes of p/T-AKT, p/T-ERK, p/T-mTOR, p/T-NF-*κ*B, and p/T-PI3K in THP-1 cells after siRNA knockdown of PRMT5 gene. (*top*) Western blot images (*β*-actin as loading control); (*bottom*) image grayscale analysis of the corresponding Western blot images in triplicates. The results suggested that the expression levels of p-ERK, p-AKT, p-NF-*κ*B, and p-mTOR were decreased in the si-PRMT5 group. All the experiments were repeated by three times. Data are expressed by mean ± standard deviation (^∗^*P* ≤ 0.05; ^∗∗^*P* ≤ 0.01; ^∗∗∗^*P* ≤ 0.001).

**Figure 7:** mTOR pathway inhibitor attenuated the migration, invasion, and adhesion of AML cells. (a) After treatment of mTOR pathway inhibitor in MV-4-11 cells for 12 h, the numbers of cell migration in the CON group and inhibitor group were detected by Transwell migration assay. (b) Quantification analysis (a) indicated that the number of cells in the inhibitor group was significantly less than that in the CON group. (c) After treatment of mTOR pathway inhibitor in MV-4-11 cells for 12 h, the numbers of cell invasion in the CON group and inhibitor group were detected by Transwell invasion assay. (d) Quantification analysis (c) indicated that the number of invasion cells in the inhibitor group was significantly less than that in the CON group. (e) After treatment of mTOR pathway inhibitor in MV-4-11 cells for 12 h, the cell adhesion was detected, and the number of adherent cells in the inhibitor group was found to be significantly less than that in the CON group. After treatment of mTOR pathway inhibitor in THP-1 for 12 h, the (f, g) migration, (h, i) invasion, and (j) adhesion of THP-1 cells were detected. The above indexes in the inhibitor group were significantly lower than those in the CON group. All the experiments were repeated by three times. Data are expressed by mean ± standard deviation (^∗^*P* ≤ 0.05; ^∗∗^*P* ≤ 0.01; ^∗∗∗^*P* ≤ 0.001). The representative images are under 100x magnification.

**Figure 8:** The effect of inhibition of PRMT5 (EPZ015666) on the expression of related genes in AML cells. (a) After treatment of MV-4-11 and THP-1 cells with PRMT5 inhibitor (EPZ015666) for 24 h, the expression of PRMT5, p/T-mTOR, and LILRB4 in the CON group and EPZ015666 group was detected by Western blot. (c) J image grayscale analysis (a) showed that PRMT5 expression was downregulated in the EPZ015666 group. (d) J image grayscale analysis (a) showed that p-mTOR expression was downregulated in the EPZ015666 group. (e) J image grayscale analysis (a) showed that LILRB4 expression was downregulated in the EPZ015666 group. *β*-Actin was used as the internal control. The same experiments and similar results were reproduced on THP-1 cells, as shown in (b) and (f–h). Data are expressed by mean ± standard deviation (^∗^*P* ≤ 0.05; ^∗∗^*P* ≤ 0.01).

**Figure 9:** The effect of inhibition of mTOR pathway on the expression of related genes in AML cells. (a) After treatment of MV-4-11 and THP-1 cells with mTOR pathway inhibitor for 12 h, the expression levels of PRMT5, p/T-mTOR, and LILRB4 in the CON group, si-CN group, si-PRMT5, and mTOR inhibitor-3 group were detected by Western blot. (b) J image grayscale analysis (a) revealed that PRMT5 had no obvious downward trend, but the expression of p-mTOR and LILRB4 was significantly decreased, and the expression of PRMT5, p-mTOR, and LILRB4 was significantly decreased in the si-PRMT5 group. *β*-Actin was used as the loading control. The same experiments and similar results were reproduced on THP-1 cells, as shown in (c, d). Data are expressed by mean ± standard deviation (^∗^*P* ≤ 0.05; ^∗∗^*P* ≤ 0.01).

**Table 1:** The characteristics of the AML patients.

Patients	Sex	Age (years)	BM/PB	FAB	WBC (10^9^L)	HB (g/L)	PLT (10^9^L)	%blasts (BM)	Evaluation
AML1	M	50	BM	M5	145.19	60	17	67.92	Initial
AML2	F	51	BM	M4	1.89	85	10	46	Initial
AML3	M	53	BM	M5	10.11	80	65	43	Initial
AML4	F	61	BM	M5	2.51	61	183	73	Initial
AML5	F	73	BM	M5	17.68	80	80	26	Initial
AML6	F	42	BM	M5	4.76	123	108	87	Relapse
AML7	M	35	BM	M4	8.68	84	21	58.6	Relapse
AML8	F	50	BM	M5	1.27	51	34	89	Initial
AML9	M	73	BM	M4	1.21	59	44	31	Initial
AML10	F	39	BM	M5	36.05	106	23	39	Initial
AML11	F	77	BM	M5	196.96	77	32	91	Initial
AML12	F	22	BM	M5	39.9	97	180	84	Relapse
AML13	M	59	BM	M5	1.97	128	91	57	Initial
AML14	F	49	BM	M5	1.3	57	113	93	Relapse
AML15	F	61	BM	M5	25.5	56	20	39	Initial
AML16	M	53	BM	M5	66.12	71	10	80	Initial
AML17	F	66	BM	M5	4.27	119	56	21	Relapse
AML18	M	23	BM	M4	95.29	135	52	89	Initial
AML19	F	47	BM	M5	1.19	68	46	38	Initial
AML20	M	56	BM	M5	14.53	72	104	85	Relapse
AML21	F	49	BM	M5	2.05	82	21	15	Relapse
AML22	M	50	BM	M5	103.76	113	58	79	Relapse
AML23	F	73	BM	M5	19.05	26	24	14	Relapse
AML24	M	39	BM	M4	6.31	71	198	39	Initial
AML25	M	73	BM	M4	5.2	105	108	27-35	Relapse
AML26	F	21	BM	M4	127.64	74	143	23	Relapse
AML27	F	39	BM	M5	5.7	78	32	50	Relapse
AML28	M	40	BM	M4	38.36	89	11	36	Relapse
AML29	M	23	BM	M4	2.41	112	211	27	Relapse
AML30	M	59	BM	M5	0.18	61	60	54	Relapse

## Data Availability

The datasets used or analyzed in the current research can be obtained from the appropriate authors according to reasonable requirements.

## References

[1] Short N. J., Rytting M. E., Cortes J. E. (2018). Acute myeloid leukaemia. *The Lancet*.

[2] Shlush L. I., Mitchell A., Heisler L. (2017). Tracing the origins of relapse in acute myeloid leukaemia to stem cells. *Nature*.

[3] Rossignol J., Polivka L., Maouche-Chretien L., Frenzel L., Dubreuil P., Hermine O. (2019). Recent advances in the understanding and therapeutic management of mastocytosis. *F1000Research*.

[4] The Cancer Genome Atlas Research Network (2013). Genomic and epigenomic landscapes of adult de novo acute myeloid leukemia. *New England Journal of Medicine*.

[5] Kayser S., Levis M. J. (2018). Advances in targeted therapy for acute myeloid leukaemia. *British Journal of Haematology*.

[6] Burnett A. K. (2012). Treatment of acute myeloid leukemia: are we making progress?. *Hematology*.

[7] Kantarjian H. (2016). Acute myeloid leukemia--major progress over four decades and glimpses into the future. *American Journal of Hematology*.

[8] Bose P., Grant S. (2015). Rational combinations of targeted agents in AML. *Journal of Clinical Medicine*.

[9] Bedford M. T., Clarke S. G. (2009). Protein arginine methylation in mammals: who, what, and why. *Molecular Cell*.

[10] Hamard P. J., Santiago G. E., Liu F. (2018). PRMT5 Regulates DNA Repair by Controlling the Alternative Splicing of Histone- Modifying Enzymes. *Cell Reports*.

[11] Tan D. Q., Li Y., Yang C. (2019). PRMT5 modulates splicing for genome integrity and preserves proteostasis of hematopoietic stem cells. *Cell Reports*.

[12] Litzler L. C., Zahn A., Meli A. P. (2019). PRMT5 is essential for B cell development and germinal center dynamics. *Nature Communications*.

[13] Liu J., Liu Y., Shao J. (2019). Zeb1 is important for proper cleavage plane orientation of dividing progenitors and neuronal migration in the mouse neocortex. *Cell Death & Differentiation*.

[14] Amano Y., Matsubara D., Yoshimoto T. (2018). Expression of protein arginine methyltransferase-5 in oral squamous cell carcinoma and its significance in epithelial-to-mesenchymal transition. *Pathology International*.

[15] Yang C. Y., Chiu L. L., Chang C. C., Chuang H. C., Tan T. H. (2018). Induction of DUSP14 ubiquitination by PRMT5-mediated arginine methylation. *The FASEB Journal*.

[16] Blanc R. S., Richard S. (2017). Arginine methylation: the coming of age. *Molecular Cell*.

[17] Richters A. (2017). Targeting protein arginine methyltransferase 5 in disease. *Future Medicinal Chemistry*.

[18] Kaushik S., Liu F., Veazey K. J. (2018). Genetic deletion or small-molecule inhibition of the arginine methyltransferase PRMT5 exhibit anti-tumoral activity in mouse models of *MLL* -rearranged AML. *Leukemia*.

[19] Strobl C. D., Schaffer S., Haug T. (2020). Selective PRMT5 inhibitors suppress human CD8(+) T cells by upregulation of p53 and impairment of the AKT pathway similar to the tumor metabolite MTA. *Molecular Cancer Therapeutics*.

[20] Yang Y., Bedford M. T. (2013). Protein arginine methyltransferases and cancer. *Nature Reviews Cancer*.

[21] Radzisheuskaya A., Shliaha P. V., Grinev V. (2019). PRMT5 methylome profiling uncovers a direct link to splicing regulation in acute myeloid leukemia. *Nature Structural & Molecular Biology*.

[22] Webb L. M., Narvaez Miranda J., Amici S. A., Sengupta S., Nagy G., Guerau-de-Arellano M. (2019). NF-kappaB/mTOR/MYC axis drives PRMT5 protein induction after T cell activation via transcriptional and non-transcriptional mechanisms. *Frontiers in Immunology*.

[23] Cheng H., Mohammed F., Nam G. (2011). Crystal structure of leukocyte Ig-like receptor LILRB4 (ILT3/LIR-5/CD85k): a myeloid inhibitory receptor involved in immune tolerance. *Journal of Biological Chemistry*.

[24] Kang X., Kim J., Deng M. (2016). Inhibitory leukocyte immunoglobulin-like receptors: immune checkpoint proteins and tumor sustaining factors. *Cell Cycle*.

[25] Hirayasu K., Arase H. (2015). Functional and genetic diversity of leukocyte immunoglobulin-like receptor and implication for disease associations. *Journal of Human Genetics*.

[26] Gui X., Deng M., Song H. (2019). Disrupting LILRB4/APOE interaction by an efficacious humanized antibody reverses T-cell suppression and blocks AML development. *Cancer Immunology Research*.

[27] Hobo W., Hutten T. J. A., Schaap N. P. M., Dolstra H. (2018). Immune checkpoint molecules in acute myeloid leukaemia: managing the double-edged sword. *British Journal of Haematology*.

[28] John S., Chen H., Deng M. (2018). A novel anti-LILRB4 CAR-T cell for the treatment of monocytic AML. *Molecular Therapy*.

[29] Deng M., Gui X., Kim J. (2018). LILRB4 signalling in leukaemia cells mediates T cell suppression and tumour infiltration. *Nature*.

[30] Dobrowolska H., Gill K. Z., Serban G. (2013). Expression of immune inhibitory receptor ILT3 in acute myeloid leukemia with monocytic differentiation. *Cytometry B Clin Cytom*.

[31] Li Z., Deng M., Huang F. (2020). LILRB4 ITIMs mediate the T cell suppression and infiltration of acute myeloid leukemia cells. *Cellular & Molecular Immunology*.

[32] Hsu J. M., Chen C. T., Chou C. K. (2011). Crosstalk between Arg 1175 methylation and Tyr 1173 phosphorylation negatively modulates EGFR-mediated ERK activation. *Nature Cell Biology*.

[33] Lu Y., Jiang Z., Dai H. (2018). Hepatic leukocyte immunoglobulin-like receptor B4 (LILRB4) attenuates nonalcoholic fatty liver disease via SHP1-TRAF6 pathway. *Hepatology*.

[34] Wei T.-Y. W., Juan C.-C., Hisa J.-Y. (2012). Protein arginine methyltransferase 5 is a potential oncoprotein that upregulates G1 cyclins/cyclin-dependent kinases and the phosphoinositide 3-kinase/AKT signaling cascade. *Cancer Science*.

[35] Zhang B., Dong S., Zhu R. (2015). Targeting protein arginine methyltransferase 5 inhibits colorectal cancer growth by decreasing arginine methylation of eIF4E and FGFR3. *Oncotarget*.

[36] Kanamaluru D., Xiao Z., Fang S. (2011). Arginine methylation by PRMT5 at a naturally occurring mutation site is critical for liver metabolic regulation by small heterodimer partner. *Molecular and Cellular Biology*.

[37] Karkhanis V., Hu Y. J., Baiocchi R. A., Imbalzano A. N., Sif S. (2011). Versatility of PRMT5-induced methylation in growth control and development. *Trends in Biochemical Sciences*.

[38] Zakrzewicz D., Didiasova M., Krüger M. (2018). Protein arginine methyltransferase 5 mediates enolase-1 cell surface trafficking in human lung adenocarcinoma cells. *Biochimica et Biophysica Acta (BBA) - Molecular Basis of Disease*.

